The article "Estrogen Replacement Therapy Induces Antioxidant and Longevity-Related Genes in Women after Medically Induced Menopause" was published in 2021. Journal: Oxid Med Cell Longev.

# Estrogen Replacement Therapy Induces Antioxidant and Longevity-Related Genes in Women after Medically Induced Menopause

**DOI:** 10.1155/2021/8101615

**Published:** 2021-09-09

**Authors:** C. Borrás, M. Ferrando, M. Inglés, J. Gambini, R. Lopez-Grueso, R. Edo, C. Mas-Bargues, A. Pellicer, J. Viña

**Affiliations:** ^1^Freshage Research Group, Department of Physiology, Faculty of Medicine, University of Valencia, CIBERFES, Institute of Health Research-INCLIVA, Avenida Blasco Ibañez no 15, 46010 Valencia, Spain; ^2^IVI-RMA Bilbao, 48940 Leioa, Spain; ^3^Freshage Research Group-Department of Physiotherapy, Faculty of Physiotherapy, University of Valencia, CIBERFES, INCLIVA, Calle Gascó Oliag no 5, 46010 Valencia, Spain; ^4^IVI-RMA Rome Parioli, 00197 Rome, Italy; ^5^Department of OB/Gyn Faculty of Medicine, University of Valencia, 46010 Valencia, Spain; ^6^Reproductive Medicine Research Group, IIS La Fe, 46026 Valencia, Spain

## Abstract

Females live longer than males in many species, including humans, and estrogens are in part responsible for this protection against aging. We reported previously that estrogens can protect rats against oxidative stress, by inducing antioxidant and longevity-related genes. Thus, this study was aimed at confirming the ability of estrogens to upregulate antioxidant and longevity-related genes in humans. For this purpose, we selected 16 women of reproductive age (18-42 years old) undergoing a fertility treatment that includes a medically induced menopause, at the Valencian Infertility Institute. We took blood samples at each time point of the treatment (basal, induced menopause, estrogen, and estrogen plus progesterone replacement therapy). mRNA expression of antioxidant and longevity-related genes in peripheral blood mononuclear cells (PBMC) was determined by real-time reverse transcriptase-polymerase chain reaction (RT-PCR). Determination of reduced glutathione (GSH) in total blood was carried out using high-performance liquid chromatography (HPLC). As expected, we found that medically induced menopause significantly decreased sexual hormone (estrogens and progesterone) levels. It also lowered glutathione peroxidase (GPx), 16S rRNA, P21, and TERF2 mRNA expression and blood GSH levels. Estrogen replacement therapy significantly restored estrogen levels and induced mRNA expression of manganese superoxide dismutase (MnSOD), GPx, 16S rRNA, P53, P21, and TERF2 and restored blood GSH levels. Progesterone replacement therapy induced a significant increase in MnSOD, P53, sestrin 2 (SENS2), and TERF2 mRNA expression when compared to basal conditions. These findings provide evidence for estrogen beneficial effects in upregulating antioxidant and longevity-related genes in women.

The article "Estrogen Replacement Therapy Induces Antioxidant and Longevity-Related Genes in Women after Medically Induced Menopause" was published in 2021. Journal: Oxid Med Cell Longev.

## 1. Introduction

The great increase in average life expectancy during the 20^th^ century emerges as one of society's greatest achievements. As a matter of fact, in the last two decades, life expectancy at birth has increased by 5–10 years [1]. Regardless of the cultural or socioeconomic context, women have lived longer than men in different countries and in every era [2]. Nowadays, 75% and 90% of people older than 100 years and 110 years (respectively) are women, and the longest living centenarian person (122 years old) was a woman. This phenomenon occurs not only in humans, but in many species, like all Old-World monkeys, apes, short-finned pilot whales, African lions, red deer and Wistar rats, in which female life expectancy exceeds male life expectancy by 16% [3, 4].

One plausible explanation for this protection against aging is that females are endowed with higher levels of estrogens than males. Estrogens are known to have many beneficial effects: cardioprotection [5], skeletal homeostasis maintenance [6], brain function [7, 8], and hematopoietic stem cell division enhancement [9], among others. Moreover, intramuscular estrogen levels have been recently associated with skeletal muscle strength and power [10]. Furthermore, they act as antioxidants *in vitro* [11] and also have beneficial effects against oxidative stress *in vivo* [4, 12]. Indeed, a few years ago, we reported that estrogens were able to induce antioxidant and longevity-related genes, such as glutathione peroxidase (GPx) and Mn-superoxide dismutase (Mn-SOD) in rats [4], through a mechanism involving the ERK1–2/NF*κ*B pathway [13]. We thus suggested that this finding could explain why females suffer less oxidative stress than males in many species, including humans [14, 15].

However, all these estrogen beneficial effects may be lost in menopause. Indeed, we observed that when mimicking postmenopausal loss of estrogens by ovariectomizing Wistar rats, their peroxide production rose, and their glutathione levels decreased. They were restored after estrogen replacement therapy [4]. This confirmed the impact of estrogen as a causative agent for this effect and made us hypothesize that this finding could be extrapolated to humans, that is, that estrogen replacement therapy (ERT) may be useful to restore estrogen levels and thus the estrogen-related beneficial effects.

Thus, the aim of this study was to confirm the ability of estrogens to upregulate antioxidant and longevity-related genes in humans, particularly in women, after a medically induced menopause. We report that ERT restores sexual hormone levels in women of reproductive age and induces the expression of antioxidant and longevity-related genes. These findings provide evidence for the beneficial antioxidant effects of estrogens in women, providing evidence that our previous studies in rodents can be translated to humans.

The article "Estrogen Replacement Therapy Induces Antioxidant and Longevity-Related Genes in Women after Medically Induced Menopause" was published in 2021. Journal: Oxid Med Cell Longev.

## 2. Materials and Methods

### 2.1. Participants and General Procedure

We recruited 16 women of reproductive age (18-42 years old) with regular cycles undergoing fertility treatment at the Valencian Infertility Institute. Causes of infertility and physiological conditions of all women were similar (i.e., hormonal alterations). Exclusion criteria were the following: vitamin supplement intake; practice of strenuous exercise; smoking; diabetes; chronic inflammatory diseases such as inflammatory bowel disease, Crohn's disease, rheumatoid arthritis or bacterial/viral pneumonia, and presence of neoplasms; and not signing the informed consent document.

Women were administered the normal therapy used in assisted reproduction cycles for oocyte donation and transfer of thawed embryos. In brief, patients received ERT using a Gonadotropin-releasing hormone agonist depot (GnRH-a) (Decapeptyl 3.75, IPSEN, France) injected on days 19-21 of the previous cycle, in the late luteal phase. Estrogen replacement was administered when the next period started, once adrenal suppression was confirmed by ultrasound examination. After 14 days of administering 6 mg/day of estradiol valerate orally (Progynova®; Schering, Spain), blood tests for hormone determination were performed. Then, patients received also micronized progesterone (800 mg/day) administered vaginally for 5 days (Progeffik®; Effik Laboratories, Madrid, Spain).

All subjects were informed verbally and in writing about the nature of this study, including all potential risks. Written informed consent was obtained prior to participation. All procedures were conducted in accordance with the principles of the World Medical Association's Declaration of Helsinki, and the protocols were approved by the Ethics Committee of the Valencian Infertility Institute (0806-C-049-SS).

### 2.2. Sampling

Blood samples were drawn from the antecubital vein at four different moments: at the beginning of the study, when women were in the late luteal phase (basal), when the next period started, i.e., 9-12 days after GnRh treatment (menopause), 14 days after estradiol treatment (estradiol), and 5 days after estradiol plus progesterone treatment (progesterone). They were collected in tubes containing heparin as anticoagulant (total blood for GSH); ethylenediaminetetraacetic acid (EDTA) as anticoagulant, in order to obtain plasma; or in VACUTAINER® CPT™ (Cell Preparation Tube) (BD, Franklin Lakes, NJ) containing sodium heparin as anticoagulant, in order to obtain peripheral blood mononuclear cells (PBMCs). For plasma isolation, EDTA-containing tubes were centrifugated at 1500 × g for 15 minutes at room temperature. For PBMC collection, VACUTAINER® CPT™ tubes were centrifuged at 3000 × g for 15 minutes at room temperature within half an hour of blood collection. We then collected the white ring containing mononuclear cells. Samples were frozen at −80°C until analysis. Laboratory personnel were all blinded to the sample's identity.

The article "Estrogen Replacement Therapy Induces Antioxidant and Longevity-Related Genes in Women after Medically Induced Menopause" was published in 2021. Journal: Oxid Med Cell Longev.

### 2.3. Determination of Reduced Glutathione (GSH) in Total Blood

Determination of reduced glutathione (GSH) was carried out using high-performance liquid chromatography with UV-visible detection, which we developed to measure GSSG in the presence of a large excess of GSH [16]. In essence, this method consists of minimizing GSH oxidation, which otherwise would result in a large increase in GSSG by using N-ethylmaleimide (NEM). In order to measure GSH, 0.5 mL of total blood was treated at 4°C with 0.5 mL ice-cold perchloric acid (6%), containing 1 mM bathophenanthroline disulphonic acid (BPDS). Samples were then centrifuged at 15,000 × g for 15 min (4°C), and the acidic supernatants were further used for total GSH determination.

### 2.4. RNA Isolation by TRIzol® and Reverse Transcription

Total RNA was isolated from PBMCs by using TRIzol® Reagent (Invitrogen™), according to the manufacturer's instructions. RNA was quantified by measuring the absorbance at 260 nm. The purity of the RNA samples was assessed by the 260/280 ratio. cDNA was then synthesized from 1000 ng total RNA by using a MultiScribe reverse transcriptase (RT) system kit (High-Capacity cDNA Reverse Transcription Kit, Applied Biosystems). As recommended by the manufacturer, the reaction was run for 10 min at 25°C, 120 min at 37°C, and 5 min at 85°C, then cooled to 4°C to collect the cDNA and finally stored at -20°C prior to the mRNA expression assays.

### 2.5. MassARRAY Quantitative Gene Expression (QGE) Analysis

According to previous experiments from our laboratory [17], cDNA was diluted 1/10 in water and 1 *μ*L of this dilution along with a synthetic competitor that had a SNP mismatch served as templates for the competitive PCR that occurs in the MassARRAY Quantitative Gene Expression (QGE) protocol. PCR products were purified with shrimp alkaline phosphatase to remove excess dNTPs. Then, they were used for an extension reaction with a cocktail of extension primers and “ACT” termination mix, containing ThermoSequenase™; dideoxynucleotide triphosphates ddATP, ddCTP, and ddTTP; and the deoxynucleotide triphosphate dGTP as included in the kit “iPLEX Gold” (Sequenom Labcorp, San Diego, CA) according to the supplier protocol. The final extension products were treated with SpectroCLEAN resin (Sequenom Labcorp, San Diego, CA) to remove salts present in the reaction buffer, and 25 *μ*L of reaction solution was dispensed onto a 384-format SpectroCHIP™, where RNA quantification was undertaken. This analysis allows the estimation of the proportion of extension products corresponding to each different gene. Therefore, the absolute molecule number was calculated for each of the PCR templates. All peaks were “called” and analysed by MassARRAY Quantitative Gene Expression 3.4 software (Sequenom Labcorp, San Diego, CA).

The article "Estrogen Replacement Therapy Induces Antioxidant and Longevity-Related Genes in Women after Medically Induced Menopause" was published in 2021. Journal: Oxid Med Cell Longev.

Multiplexed primer and competitive template designs were created using the MassARRAY QGE Assay Design software v1.0 (Sequenom, Labcorp, San Diego, CA) for random hexamer priming, such that at least one PCR primer spanned an exonic boundary per each transcript assayed.

Copy number determination for each transcript was conducted using real-time competitive PCR coupled with product resolution via Matrix-Assisted Laser Desorption/Ionization Mass Spectrometry (MassARRAY QGE, Sequenom, Labcorp, San Diego, CA), as previously described [18]. Products were resolved on a linear MALDI-TOF mass spectrometer (MassARRAY Compact, Sequenom, Labcorp, San Diego, CA). Signal acquisition, allele assignment, and peak area integration per spectrum were conducted with the MassARRAY RT Workstation v3.4 (Sequenom, Labcorp, San Diego, CA). Data was analysed using MassARRAY QGE Analyzer v3.4 (Sequenom, Labcorp, San Diego, CA) with copy numbers for each transcript per sample determined based on the EC50 of standard curve titrations of known competitor amounts per assay vs. a fixed amount of cDNA template.

Normalization of copy numbers between samples for the different assays was conducted using a multiplexed set of 3 well-characterized human housekeeping (normalization) transcripts (ACTB-6, GAPDH-6, and HMBS-7) and geNorm software. Normalization factors per sample were calculated using the geometric mean of the most stable combination of these normalization assays, determined by the measure of their pairwise variation as calculated by geNorm [19].

### 2.6. mRNA Gene Expression by Real-Time Polymerase Chain Reaction (RT-PCR)

mRNA expression of those genes that were not initially included in the MassARRAY assays were determined by real-time PCR with glyceraldehyde-3P-dehydrogenase (GAPDH) as the endogenous control, according to previously published results [13, 20]. For this purpose, a quantitative PCR was performed using the detection system 7900HT Fast Real-Time PCR System (Applied Biosystems) and Maxima® SYBR Green/ROX qPCR Master Mix (2X) (Fermentas). Target and control genes were run in triplicate as follows: 10 min at 95°C and then 35 cycles of: denaturation for 15 s (95°C) and annealing and extension for 1 min (62°C). Specific primers were employed for each gene. The threshold cycle (CT) was determined, and then, the relative gene expression was analyzed using the standard curve method.

The article "Estrogen Replacement Therapy Induces Antioxidant and Longevity-Related Genes in Women after Medically Induced Menopause" was published in 2021. Journal: Oxid Med Cell Longev.

### 2.7. Statistical Analysis

Standard statistical methods were used to obtain the mean and standard deviation of the mean (SD). After checking the normality of the variables with the Shapiro-Wilk test (*p* > 0.05), a repeated measure of analysis of variance (ANOVA) with Bonferroni post hoc was used for the comparison of each variable between the different treatment times. The type I error was established as < 5% (*p* < 0.05). All statistical analyses were performed with SPSS v.22 (IBM SPSS, Inc., Chicago, IL, USA).

## 3. Results

### 3.1. ERT Restores Sex Hormone Levels after GnRH-a-Induced Menopause

Menopause is known to decrease sex hormone levels, thus producing negative outcomes. Indeed, we found a decrease in estrogens (*p* < 0.01) and progesterone (*p* < 0.01) levels in women after 10 days of GnRH-a treatment, when compared to basal levels (Figures 1(a) and 1(b)). After 14 days of administering 6 mg/day of estradiol valerate orally, estrogen levels increased significantly compared to menopause (*p* < 0.01) and even basal (*p* < 0.01) levels (Figure 1(a)). At this point, progesterone levels remained low, compared to basal levels (*p* < 0.01) (Figure 1(b)). After 5 days of treatment with progesterone, its levels returned to basal (Figure 1(b)). These results confirm the restoration of sex hormone levels caused by ERT after GnRH-a-induced menopause.

### 3.2. ERT Acts as an Antioxidant in Menopausal Women

Previous data from our laboratory suggest that female rats may live longer than males due to the protective effect of estrogens, which are able to act as an antioxidant by upregulating antioxidant genes [4, 13], but these effects had not been tested in humans. Women after GnRH-a-induced menopause showed reduced blood glutathione levels (*p* < 0.05 compared to basal levels) which were restored by ERT (*p* < 0.05 compared to menopause levels). Progesterone administration did not show any effect (Figure 2(a)).

Moreover, as shown in Figure 2(b), estrogen and progesterone administration after a medically induced menopause was able to increase MnSOD expression (*p* < 0.05 compared to basal). GPx mRNA levels, which were downregulated after menopause (*p* < 0.05 compared to basal), returned to basal levels (*p* < 0.05 compared to menopause). Progesterone administration did not show any effect in this case either (Figure 2(c)).

The article "Estrogen Replacement Therapy Induces Antioxidant and Longevity-Related Genes in Women after Medically Induced Menopause" was published in 2021. Journal: Oxid Med Cell Longev.

Thus, we have found that the upregulation of antioxidant genes by estradiol can be translated to humans.

### 3.3. ERT Upregulates the Expression of the Longevity-Related Gene 16S Ribosomal RNA (16S rRNA) in Women after a Medically Induced Menopause

Expression of 16S rRNA decreases significantly under conditions of oxidative stress [21] and also with aging [22]; thus, it could be considered as a longevity-related gene. We previously reported that female rats overexpressed this mitochondrial rRNA subunit when compared with males. Here, we found that 16S rRNA expression was diminished after menopause (*p* < 0.05 compared to basal levels) and increased significantly after estrogen administration (*p* < 0.05 compared to menopause levels), thus confirming our previous results in humans. Progesterone administration did not show any effect (Figure 3).

### 3.4. ERT Increases Other Longevity-Related Pathways in Women after GnRH-a-Induced Menopause

P53 is known to possess both an anticancer and antiaging effect [23]. In this regard, we studied P53 mRNA expression by RT-PCR in women who underwent a medically induced menopause. Interestingly, we found that ERT resulted in an increase in P53 mRNA levels after 14-day estradiol treatment (*p* < 0.01) and remained high 5 days after progesterone treatment (*p* < 0.01), comparing to basal levels (Figure 4(a)).

P21 constitutes a crucial target of P53, and its upregulation leads to G1 arrest following P53 activation by stress stimuli [24]. Noteworthy, we found that P21 mRNA levels decreased in our menopause model (*p* < 0.05 compared to basal levels) but returned to basal levels after 14 days of estradiol administration (*p* < 0.05 compared to menopause levels) (Figure 4(b)).

In addition to its antioxidant activity, Sestrin-2 (SESN2) is closely linked to P53 expression [25–27]. We found that estradiol and progesterone administration after menopause increased SENS2 mRNA levels (Figure 4(c), *p* < 0.05 compared to basal; *p* < 0.05 compared to menopause levels).

Another longevity-related gene linked to P53 is the telomeric repeat binding factor 2 (TERF2). TERF2 is located in the shelterin complex that protects the telomeres from degradation and inappropriate DNA repair and prevents end-to-end fusion, atypical recombination, and premature senescence [28]. P53, a downstream effector of the telomere damage signaling, also functions upstream of the telomere-capping protein complex by inducing TERF2 protein degradation, which can be a signal for enhancing gene expression of this protein [29]. As shown in Figure 4(d), we found that decreased TERF2 mRNA expression after medically induced menopause was restored by estrogen administration (*p* < 0.01) and remained high 5 days after progesterone treatment (*p* < 0.01), when compared to the basal point.

The article "Estrogen Replacement Therapy Induces Antioxidant and Longevity-Related Genes in Women after Medically Induced Menopause" was published in 2021. Journal: Oxid Med Cell Longev.

## 4. Discussion

The current study shows that ERT restores sexual hormone levels and induces the expression of antioxidant and longevity-related genes in women of reproductive age undergoing a medically induced menopause. To the best of our knowledge, this is the first study to evaluate the beneficial antioxidant effects of ERT in women of reproductive age undergoing a transient menopause.

GnRH-a therapy is commonly practiced as an infertility treatment. It decreases the production of estrogens to the levels women have after menopause, so this human model of estrogen deprivation can be considered as a model of transient menopause that allows the study of the biological effects of estrogen deficiency and subsequent reposition [30]. Moreover, inclusion of young premenopausal women eliminates confounding factors, such as chronic diseases, which may underestimate the magnitude of the effect of estrogens on antioxidant and longevity-related genes.

A growing body of research on sex differences in mortality across species supports that females live longer than men in many species, including humans [2, 4, 31]. Although this is not a universal phenomenon (i.e., in some species, females and males display the same average lifespan or males even live longer than females [3]), the general claim is that the survival advantage of females is fundamentally due to biological factors, rather than environmental or social factors. Indeed, females survive better than males under extreme conditions (i.e., famines, epidemics) and even during childhood, when social and environmental just differences may be minimal or even favor males [32]. Among these biological factors, the beneficial effects of estrogens beyond their pivotal role in sexual development and reproduction have been well documented [5–10]. However, in rodents such as mice, some strains show no differences in longevity between sexes [33], which is against the protective role of estrogens on longevity. These are inbred strains, which probably during this inbred process have suffered changes in hormonal sensitivity [34].

Besides sex, age and hormones are important factors to consider when referring to the antioxidant status. Regarding the former, the “free radical theory of aging” postulates that the loss of balance between prooxidants and antioxidants leads to accumulation of oxidative damage in macromolecules with age, which plays an important role in age-related disturbances in cellular processes [35]. In this regard, an impairment of the antioxidant status has been reported with age in humans [36, 37]. However, these studies have included age groups over 55 years old or even have considered individuals under 55 as a control group. According to these findings, the antioxidant status in the age group included in our study (i.e., under 40) is similar. Furthermore, women under 40 years old are endowed with female hormones (i.e., estrogens and progesterone), which confers them protection against oxidative damage.

The article "Estrogen Replacement Therapy Induces Antioxidant and Longevity-Related Genes in Women after Medically Induced Menopause" was published in 2021. Journal: Oxid Med Cell Longev.

Indeed, our results support the favorable effects of estrogens, since we found that in women of reproductive age, when they are medically deprived of estrogens, they display decreased blood GSH levels and downregulate antioxidant (GPx, MnSOD, and SENS2) and longevity-related (16S rRNA, P53, P21, and TERF2) genes. Interestingly, when estrogen levels are restored by means of ERT, all these effects are counteracted or even improved, indicating that ERT act as an antioxidant in women. This is in agreement with our previous work showing that female rats (endowed with higher blood GSH levels and higher GPx, Mn-SOD, and 16S rRNA mRNA levels than men) undergoing ovariectomy (a model of menopause in animals) showed an increased peroxide production caused by a decrease in blood GSH levels, and they downregulated GPx and Mn-SOD gene expression [4]. Afterwards, when estrogens were restored, all these variables were improved to normal levels, thus confirming that estrogens were responsible for these detrimental effects, through a mechanism involving the ERK1–2/NF*κ*B pathway [13]. In humans, similar results have been found in a model of surgical estrogen deprivation, where women undergoing bilateral oophorectomy displayed increased oxidative stress (i.e., an increase in GSSG/GSH ratio and a reduction in MnSOD and GPx mRNA gene expression), which was completely restored after ERT [38]. Taken together, these results make us hypothesize that ERT is able to restore antioxidant status by activating the ERK1–2/NF*κ*B pathway, thus resulting in the upregulation of antioxidant genes.

Classically, estrogens bind to their specific estrogen receptor (Er*α*, Er*β*) to exert its genomic regulatory effects. As ligand-dependent transcriptional factors, the hormone-bound estrogen receptors interact with estrogen response elements (ERE) to stimulate several genes in estrogen-responsive tissues and to regulate gene transactivation [39]. However, around one-third of the human genes that are regulated by estrogens do not contain ERE-like sequences, like Mn-SOD and GPx [40]. Thus, activation of target genes by estrogens may also be mediated by other transcription factors, including AP-1 and NF-*κ*B, independent of the ERE [41]. Here, we hypothesize, according to our previous results [13] and to other authors [38], that estrogen replacement therapy is able to restore antioxidant status by activating the ERK1–2/NF*κ*B pathway, which in turn upregulates antioxidant genes. Other proposed mechanisms of estrogens that may influence ERT beneficial effects include modulation of vascular function and inflammatory response as well as metabolic and hemodynamic effects [42]. This may be due to estrogen ability to increase eNOS and antioxidant gene expression in the vasculature and other tissues, resulting in reduced oxidative stress and increased NO bioavailability, and the modulation of the renin-angiotensin system [42]. Furthermore, a recent review found that ERT significantly decreases the risk of onset and/or development of AD, thus highlighting the neuroprotective role of this therapy, through a variety of mechanisms (reviewed in [43]).

The article "Estrogen Replacement Therapy Induces Antioxidant and Longevity-Related Genes in Women after Medically Induced Menopause" was published in 2021. Journal: Oxid Med Cell Longev.

ERT has been widely used to restore the beneficial effects of menopause, but its potentially detrimental role has been a matter of controversy for several years. However, when HRT is not administered immediately after menopause, estrogen favorable effects may disappear [44–47]. We recently provided evidence supporting this hypothesis and found that estrogen deprivation in ovariectomized rats caused oxidative stress that was prevented by HRT only if started immediately after ovariectomy [48].

Finally, our results support the notion that sex differences in the antioxidant system are extremely important to consider, especially in the pathophysiology of aging and chronic diseases. In this regard, it is necessary that future research uncovers steroid hormone (i.e., estrogen, progesterone, and testosterone) actions, while encompassing other aspects including environmental and genetic factors. All these factors should be further evaluated as therapeutic targets for age-related diseases, especially those that exhibit clear gender differences, like Alzheimer's disease.

## 5. Conclusion

ERT induces antioxidant and longevity-related genes in women of reproductive age after medically induced menopause. These findings confirm the translationality of our previous results in rodents and may provide evidence on the biological factors contributing to the longer lifespan in women.

## Figures and Tables

**Figure 1:** ERT restores plasma estrogen levels (a) and plasma progesterone levels (b) in women of reproductive age who underwent GnRH-a-induced menopause. Data are expressed as median and range with 95% CI for 16 women at four different blood sampling times: basal, menopause (after 10 days of GnRH-a treatment), estrogens (after 14 days 6 mg estradiol treatment), and progesterone (after 5 days of 800 mg progesterone treatment).

The article "Estrogen Replacement Therapy Induces Antioxidant and Longevity-Related Genes in Women after Medically Induced Menopause" was published in 2021. Journal: Oxid Med Cell Longev.

**Figure 2:** (a) ERT restores plasma GSH levels after pharmacological-induced menopause. (b) MnSOD and (c) GPx mRNA levels increase after ERT in women of reproductive age who underwent GnRH-induced menopause. Data are expressed as median and range with 95% CI for 16 women of reproductive age who underwent GnRH-induced menopause.

**Figure 3:** ERT increases 16S rRNA gene expression to basal levels after GnRH-induced menopause. Data are expressed as median and range with 95% CI for 16 women of reproductive age who underwent GnRH-induced menopause.

**Figure 4:** (a) ERT after GnRH-induced menopause upregulates TP53 gene expression. (b) ERT restores basal levels of P21 gene expression after pharmacological-induced menopause. (c) SESN2 mRNA levels increase after ERT in 16 women of reproductive age who underwent GnRH-induced menopause. (d) ERT restores TERF2 mRNA levels after GnRH-induced menopause. Data are expressed as median and range with 95% CI for 16 women of reproductive age who underwent GnRH-induced menopause.

## Data Availability

The data that support the findings of this study are available from the corresponding author (M. Inglés), upon reasonable request.
